The article "Innate Immune Sensing of Modified Vaccinia Virus Ankara (MVA) Is Mediated by TLR2-TLR6, MDA-5 and the NALP3 Inflammasome" was retracted in 2022. Reasons: duplicated images; unreliable images; unreliable results or conclusions; concerns about the images.

# Innate Immune Sensing of Modified Vaccinia Virus Ankara (MVA) Is Mediated by TLR2-TLR6, MDA-5 and the NALP3 Inflammasome

**DOI:** 10.1371/journal.ppat.1000480

**Published:** 2009-06-19

**Authors:** Julie Delaloye, Thierry Roger, Quynh-Giao Steiner-Tardivel, Didier Le Roy, Marlies Knaup Reymond, Shizuo Akira, Virginie Petrilli, Carmen E. Gomez, Beatriz Perdiguero, Jürg Tschopp, Giuseppe Pantaleo, Mariano Esteban, Thierry Calandra

**Affiliations:** 1 Infectious Diseases Service, Department of Medicine, Centre Hospitalier Universitaire Vaudois and University of Lausanne, Lausanne, Switzerland; 2 Department of Host Defense, Research Institute for Microbial Diseases, Osaka University, Osaka, Japan; 3 Department of Biochemistry, University of Lausanne, Epalinges, Switzerland; 4 Centro Nacional de Biotecnología, CSIC, Ciudad Universitaria Cantoblanco, Madrid, Spain; 5 Laboratory of AIDS Immunopathogenesis, Immunology and Allergology Service, Department of Medicine, Centre Hospitalier Universitaire Vaudois and University of Lausanne, Lausanne, Switzerland; University of Florida, United States of America

## Abstract

Modified vaccinia virus Ankara (MVA) is an attenuated double-stranded DNA poxvirus currently developed as a vaccine vector against HIV/AIDS. Profiling of the innate immune responses induced by MVA is essential for the design of vaccine vectors and for anticipating potential adverse interactions between naturally acquired and vaccine-induced immune responses. Here we report on innate immune sensing of MVA and cytokine responses in human THP-1 cells, primary human macrophages and mouse bone marrow-derived macrophages (BMDMs). The innate immune responses elicited by MVA in human macrophages were characterized by a robust chemokine production and a fairly weak pro-inflammatory cytokine response. Analyses of the cytokine production profile of macrophages isolated from knockout mice deficient in Toll-like receptors (TLRs) or in the adapter molecules MyD88 and TRIF revealed a critical role for TLR2, TLR6 and MyD88 in the production of IFNβ-independent chemokines. MVA induced a marked up-regulation of the expression of RIG-I like receptors (RLR) and the IPS-1 adapter (also known as Cardif, MAVS or VISA). Reduced expression of RIG-I, MDA-5 and IPS-1 by shRNAs indicated that sensing of MVA by RLR and production of IFNβ and IFNβ-dependent chemokines was controlled by the MDA-5 and IPS-1 pathway in the macrophage. Crosstalk between TLR2-MyD88 and the NALP3 inflammasome was essential for expression and processing of IL-1β. Transcription of the *Il1b* gene was markedly impaired in TLR2^−/−^ and MyD88^−/−^ BMDM, whereas mature and secreted IL-1β was massively reduced in NALP3^−/−^ BMDMs or in human THP-1 macrophages with reduced expression of NALP3, ASC or caspase-1 by shRNAs. Innate immune sensing of MVA and production of chemokines, IFNβ and IL-1β by macrophages is mediated by the TLR2-TLR6-MyD88, MDA-5-IPS-1 and NALP3 inflammasome pathways. Delineation of the host response induced by MVA is critical for improving our understanding of poxvirus antiviral escape mechanisms and for designing new MVA vaccine vectors with improved immunogenicity.

## Author Summary

Modified vaccinia virus Ankara (MVA) is a highly attenuated, replication-deficient, poxvirus currently developed as a vaccine vector against a broad spectrum of infectious diseases including HIV, tuberculosis and malaria. It is well known that robust activation of innate immunity is essential to achieve an efficient vaccine response, and that poxviruses have developed numerous strategies to block the innate immune response. Yet, the precise mechanisms underlying innate immune sensing of MVA are poorly characterized. Toll-like receptors (TLR), RIG-I-like receptors (RLR) and NOD-like receptors (NLR) are families of membrane-bound and cytosolic sensors that detect the presence of microbial products and initiate host innate and adaptive immune responses. Here, we report the first comprehensive study of MVA sensing by innate immune cells, demonstrating that TLR2-TLR6-MyD88, MDA-5-IPS-1 and NALP3 inflammasome pathways play specific and coordinated roles in regulating cytokine, chemokine and interferon response to MVA poxvirus infection. Delineation of the pathways involved in the sensing of MVA by the host could help designing modified vectors with increased immunogenicity, which would be of particular importance since MVA is considered as a leading vaccine for HIV/AIDS vaccine following the recent failure of an adenovirus-mediated HIV vaccine trial.

## Introduction

Attenuated poxviruses are currently being developed as vaccines vectors against various infectious diseases including HIV, malaria and tuberculosis [1]. Modified vaccinia virus Ankara (MVA) and NYVAC are highly attenuated poxvirus strains due to multiple deletions of viral genes and are replication-deficient in human cells. MVA and NYVAC are immunogenic and safe and have been shown to be excellent vaccine vectors for the expression of foreign antigens. MVA is a leading vaccine candidate for delivery of HIV genes with efficient induction of T-cell mediated immune responses [1]–[3]. Profiling of the immune responses triggered by poxvirus vaccine vectors is critical not only for optimal design of vaccine vectors but also for anticipating potential harmful interactions between naturally acquired or vaccine-induced immune responses against the vaccine target. This is indeed an important lesson learned from the adenovirus type 5 (Ad5) HIV vaccine (MRKAd5) STEP trial. Pre-existing neutralizing antibodies against the Ad5 vaccine vector were found to increase the relative risk of HIV infection [4],[5]. Hence the need for extensive assessments of vaccine-induced innate and adaptive immune responses to prevent unexpected adverse events.

Sensing of invasive pathogens by sentinel innate immune cells is a fundamental feature of the host antimicrobial defense response. Toll-like receptors (TLRs), retinoic acid-inducible gene-I (RIG-I) like receptors (RLRs) and nucleotide-binding and oligomerization domain (NOD)-like receptors (NLRs) have recently emerged as central innate sensors of viruses [6]. Virus sensing by TLR occurs at the cell surface and in the endosomal compartment. At the cell surface, TLR2 or TLR4 recognize either DNA (herpes viruses) or RNA viruses (respiratory syncitial, hepatitis C and measles viruses). In the endosomal compartment, TLR7, TLR3 or TLR9 sense single stranded (vesicular stomatitis virus, Sendai, West Nile and influenza viruses) and double stranded (reovirus) RNA viruses, and DNA viruses (herpes simplex viruses, cytomegalovirus), respectively [7]–[13]. Two members of the cytosolic pattern recognition RLR receptors, RIG-I (also known as DDX58) and melanoma differentiation-associated gene 5 protein (MDA5) (also known as helicard), have been shown to function as sensors of RNA viruses [14]–[19]. RIG-I detects 5′-triphosphate of ssRNAs and short dsRNAs, while MDA5 preferentially recognizes long dsRNAs. NALP3 (NLRP3 also known as cryopyrin) is a member of the NLR family which have been involved in the sensing of both DNA (adenovirus) and RNA (rotavirus, Sendai and influenza viruses) viruses [20],[21]. NALP3, ASC and pro-caspase 1 form a multimeric cytosolic molecular complex known as the NALP3 inflammasome that controls the processing of the IL-1β cytokine precursor pro-IL-1β into IL-1β [22]. Sensing of viruses by TLRs, RLRs and NLRs activates intracellular signalling pathways resulting in the expression of pro-inflammatory cytokines and type I interferons that then act on innate immune cells to limit viral replication and promote the adaptive immune response.

Here we report that the TLR2-TLR6-MyD88, MDA-5-IPS-1 and NALP3 inflammasome pathways are the main innate sensors of MVA in the macrophage and that they induce a cytokine response profile characterized by a vigorous chemokine, IFNβ and IL-1β production. Beyond the dissection of the molecular bases of MVA recognition by the innate immune system the present data are likely to help design MVA vaccine vectors with improved immunogenicity.

## Results

### Innate immune responses elicited by MVA

The profile of innate immune responses elicited by MVA was first examined by RT-PCR and ELISA in a mouse model of poxvirus infection [23]. MVA infection induced a robust innate immune response in peritoneal cells, peritoneal lavage fluid, splenocytes and splenocyte homogenates characterized by the production of pro-inflammatory cytokines (TNF, IL-1β, IL-6, IL-12p40), chemokines (IP-10/CXCL10, RANTES/CCL5, MCP-5/CCL12, MIP-2/CXCL2) and type I interferon (IFNβ) mRNA and protein (Figure 1A and B and data not shown). Infection of human whole blood with MVA also induced a vigorous innate immune response characterized by an abundant production of chemokines (IL-8/CXCL8, MIP-1α/CCL3 and IP-10) and less abundant production of pro-inflammatory cytokines (TNF, IL-1β, IL-6) (Figure 2). Interestingly, MVA was previously shown to down-regulate IL-8 and IL-1β mRNA expression in human monocyte-derived dendritic cells [24],[25], suggesting that MVA infection may induce the production of various patterns of cytokine depending upon the cell-type studied.

**Figure 1:** MVA stimulates cytokine, chemokine and IFNβ production *in vivo*. BALB/c mice were injected i.p. with MVA (10^7^ PFU). Peritoneal cells (A) and peritoneal lavage fluid (B) were collected 12 h after infection as described in *Materials and Methods*. TNF, IL-1β, IL-12p40, IP-10, RANTES and IFNβ mRNA contents of peritoneal cells were analyzed by RT-PCR (A). Results are expressed as the ratio of cytokines, chemokines or IFNβ mRNA levels to that of HPRT. AU: arbitrary units. Cytokine concentrations in peritoneal lavage fluid were measured by ELISA (B). Data are means±SD of triplicate samples from one experiment comprising three mice per experimental condition and are representative of two independent experiments. *p*<0.05 for all conditions when comparing PBS versus MVA.

**Figure 2:** TNF, IL-1β, IL-6, IL-8, MIP-1α and IP-10 release by human whole blood exposed to MVA. Whole blood from 3 healthy volunteers (#1, 2 and 3) was incubated for 24 h with (+) or without (−) MVA (MOI 1) in triplicates. Cell-free supernatants were collected to quantify the concentrations of TNF, IL-1β, IL-6, IL-8, MIP-1α and IP-10. Data are means±SD of triplicate samples from one experiment. MVA significantly increased cytokine production (*p*<0.05 for all conditions).

Dissection of the molecular mechanisms of MVA-induced innate immune responses was preformed in PMA-differentiated human THP-1 macrophages and primary human macrophages. Flow cytometry analyses performed with GFP-expressing MVA (MOI 5) indicated that MVA rapidly infected THP-1 cells (Figure 3A and B). More than 60% of cells became GFP positive within 2 h followed by a progressive decline of GFP fluorescence thereafter, which could result either from MVA-induced apoptosis as observed in human HeLa and monocyte-derived dendritic cells [24],[25] or from the shutting down of protein synthesis through activation of the PKR pathway by MVA [26]. Indeed, the number of apoptotic cells increased from 5% at 6 h to 35% at 24 h post-infection as assessed by annexin V and propidium iodine staining (data not shown).

**Figure 3:** MVA induces the production of cytokines, chemokines and IFNβ by human macrophages. Human THP-1 cells (A–E) and primary human macrophages (F) were infected with GFP-positive (A, B) or wild-type (C–F) MVA (MOI 5). Expression of viral-derived GFP protein by THP-1 cells analyzed by flow cytometry (A, B). Cytokines, chemokines and IFNβ production by THP-1 cells stimulated for 24 h with MVA as assessed by the Luminex technology (C) or by ELISA (D). IL-8 (CXCL8), MIP-1α (CCL3), RANTES (CCL5), IP-10 (CXCL10) and IFNβ mRNA levels were analyzed by RT-PCR and results expressed as the ratio of chemokines or IFNβ to HPRT mRNA levels. AU: arbitrary units (E, F). Data are means±SD of duplicate (C) or triplicate (D to F) samples from one experiment and are representative of one (C) to three (D to F) independent experiments. *p*<0.05 for all conditions (D to F).

The profile of cytokines and chemokines released by MVA-infected THP-1 cells was analyzed with the Luminex technology. Twenty four h after infection, 12 of the 30 mediators analyzed (see *Materials and Methods*) were detectable in cell-culture supernatants. Similarly to the results obtained with human whole blood (Figure 2) and in agreement with a recent report by Lehmann *et al.* [27], MVA induced the production of large quantities of chemokines (IL-8, MIP-1α, MIP-1β/CCL4, MCP-1/CCL2, RANTES and IP-10). MVA also induced large amounts of IFNβ and of IL-1ra, but small amounts of pro-inflammatory cytokines (TNF, IL-1α, IL-1β, IL-6 and IL-12p40) (Figure 3C and D). Kinetics and patterns of chemokines and type I interferon mRNA expression were similar in MVA-stimulated THP-1 cells and primary human macrophages (Figure 3E and F). We then also examined the production of cytokines and chemokines induced by two other vaccinia virus (i.e. the attenuated NYVAC strain and the virulent Western Reserve strain). When compared to MVA, NYVAC induced low levels of IL-8, IL-1β and IFNβ and no TNF, IL-6, MIP-1α, RANTES or IP-10 (Figure S1). The virulent Western Reserve strain of vaccinia virus was observed to also induce low levels of IL-8 and IFNβ in THP-1 cells, but no IL-1β, MIP-1α or IP-10 (Figure S2 and data not shown).

Altogether, these results indicated that the innate immune response induced by MVA in human macrophages was characterized by a powerful chemokine production and a less abundant production of pro-inflammatory cytokines probably related to the attenuation of MVA [28]. In contrast, the NYVAC and Western reserve strains stimulated less powerful chemokine and cytokine responses, that most likely reflect differences in the expression of immunomodulatory genes in the genome of MVA, NYVAC and Western Reserve [24],[25].

### TLR2, TLR6 and MyD88 are critical for IFNβ-independent chemokine production after MVA infection

TLRs have been shown to play an important role in the sensing of viruses and in the initiation of the anti-viral host defense response [29],[30]. Analyses of the TLR repertoire used by the host for sensing of MVA were conducted in bone marrow-derived macrophages (BMDMs) isolated from TLR1^−/−^, TLR2^−/−^, TLR4^−/−^, TLR6^−/−^, MyD88^−/−^ and TRIF^−/−^ mice and the read-out was the expression of IFN-independent chemokine MIP-2 and of IFNβ. MVA-induced MIP-2 production by BMDMs was completely abrogated in TLR2^−/−^, TLR6^−/−^ and MyD88^−/−^ cells but not in TLR1^−/−^, TLR4^−/−^ and TRIF^−/−^ cells, which produced amounts of MIP-2 similar to that of wild-type cells (Figure 4A). In contrast, the amount of IFNβ produced by TLR2^−/−^, TLR6^−/−^ and MyD88^−/−^ BMDMs was similar to that of wild-type cells (Figure 4B), a finding consistent with the notion that activation of the TLR2 pathway is not implicated in the production of type I IFNs. Similar results were obtained with THP-1 cells stably transduced with a lentiviral delivery system expressing a short hairpin RNA (shRNA) targeting the expression of the *TLR2* gene (Figure S3). All together, these results indicated that the activation of the TLR2-TLR6-MyD88 pathway was required for the induction of IFNβ-independent chemokines in MVA-stimulated macrophages. Experiments conducted with NYVAC and the Western Reserve strain of vaccinia virus confirmed that TLR2 was required for IL-8 production by THP-1 cells (Figure S1 and S2).

**Figure 4:** TLR2, TLR6 and MyD88 are critical for IFNβ-independent chemokine production after MVA infection. MIP-2 (A) and IFNβ (B) produced by wild-type, TLR1^−/−^, TLR2^−/−^, TLR4^−/−^, TLR6^−/−^, MyD88^−/−^ and TRIF^−/−^ bone marrow-derived macrophages infected with MVA (MOI 5 and 20) or stimulated with lipopolysaccharide (LPS, 100 ng/ml), Pam_2_CSK_4_ (P_2_CSK_4_, 10 µg/ml), Pam_3_CSK_4_ (P_3_CSK_4_, 10 µg/ml) for 24 h. Data are means±SD of triplicate samples from one experiment and are representative of 2 to 4 experiments.

### Endocytosis is required for IL-1β and IFNβ production

Vaccinia virus penetrates into target cells either by endocytosis or by membrane fusion in a low pH-independent manner [31]. To determine the contribution of endocytosis to MVA-induced intracellular signalling and cytokine production, THP-1 cells were treated with cytochalasine D, an actin-depolymerizing drug that blocks the endocytotic trafficking, or with chloroquine, a lysosomotropic weak base to neutralize the acidic environment of endocytic vesicles. IL-1β and to a lesser extend IFNβ production were inhibited by cytochalasine D and chloroquine treatment. The inhibition was not related to drug toxicity because chloroquine did not affect IL-8 production and cell viability (Figure 5 and data not shown). The reason why the inhibition of cytokine production (particularly IFNβ) was only partial after treatment with the inhibitors remains uncertain. The data suggest that additional non-endocytic pathways may play a role in the production of IFNβ. In agreement with a key role for membrane-bound TLR2 for IL-8 induction, the production of IL-8 was not reduced after cytochalasine D or chloroquine treatment (Figure 5). UV treatment of MVA causing a nearly complete (i.e. 90%) inhibition of the expression of the early C6L gene (data not shown) did not affect IL-1β, IL-8 and IFNβ production (Figure 5). Although one cannot completely rule out a contribution of residual viral protein synthesis, these observations support the view that induction of cytokines by MVA is most likely independent of viral gene synthesis [32]–[34]. Overall, endocytosis of MVA was required for IL-1β and IFNβ release suggesting a role for intracellular pattern recognition receptors in the production of these cytokines.

**Figure 5:** Endocytosis is required for IL-1β and IFNβ production after MVA infection. THP-1 cells were preincubated for 1 h with or without cytochalasin (2 µM) or chloroquine (100 µM) prior to exposure to MVA or UV-treated MVA (MOI 20). Cell-culture supernatants were harvested after 6 h (IL-1β) or 24 h (IFNβ and IL-8) and cytokine concentrations were measured by ELISA. Data are means±SD of triplicate samples from one experiment and are representative of two independent experiments.

### MVA is sensed by MDA-5 and not by RIG-I

The RLR family of cytosolic pattern recognition receptors has been implicated in the sensing of RNA viruses [35], but very little is known about their role in host response to DNA viruses. Extending the observations by Guerra *et al.* who noted an increased expression of RIG-I and MDA-5 mRNA in human dendritic cells infected with MVA [24], we observed that MVA caused a time-dependent increase in RIG-I, MDA-5 and IPS-1 mRNA and protein expression in THP-1 cells (Figure 6A and B). RIG-I and MDA-5 mRNAs rose within 3 h of infection and remained elevated for up to 24 h (Figure 6A). *In vivo*, MVA up-regulated RIG-I and MDA-5 mRNA levels in peritoneal cells and splenocytes (Figure S4). When compared to MVA, NYVAC induced lower levels of MDA-5 and, to a lesser extent, RIG-I and IPS-1 mRNA and protein expressions (Figure S1 and data not shown). Using shRIG-I, shMDA-5 and shIPS-1 THP-1 cells (Figure S5), we then examined whether RIG-I and MDA-5 were involved in MVA-induced IFNβ production. IFNβ and IP-10 mRNA and protein levels were markedly reduced in shMDA-5 and shIPS-1 cells, but not in shRIG-I cells. By contrast, the time-course and magnitude of the IL-8 and IL-1β production was similar in shMDA-5, shIPS-1, shRIG-I and control THP-1 cells (Figure 7A and B). Sensing of MVA by the MDA-5/IPS-1 pathway is therefore critical for the production of IFNβ and IFNβ-dependent chemokines in macrophages. In line with these data, the production of IFNβ, but not of IL-8, was also dependent on the MDA-5/IPS-1 pathway in cells infected with NYVAC and the Western Reserve strain of vaccinia virus (Figure S1 and S2).

**Figure 6:** MVA up-regulates the expression of RIG-I, MDA-5 and IPS-1 mRNAs and proteins. RIG-I, MDA-5 and IPS-1 mRNA and protein expression by RT–PCR (A) and Western blot (B). THP-1 cells were infected with MVA (MOI 5) for the indicated time. Results are expressed as the ratio of RIG-I, MDA-5 or IPS-1 mRNA levels to that of HPRT. Data are means±SD of triplicate samples from one experiment and are representative of three independent experiments. AU: arbitrary units. *p<0.05.

**Figure 7:** MVA is sensed by MDA-5 and not by RIG-I. THP-1 cells stably transduced with control, MDA-5, RIG-I or IPS-1 shRNAs were infected with MVA (MOI 5 unless specified otherwise) for the indicated time. IFNβ, IP-10, IL-8 and IL-1β mRNA and protein expression by RT-PCR and ELISA (A–B). Results are expressed as the ratio of IFNβ, IP-10, IL-8 or IL-1β mRNA levels to that of HPRT. Data are means±SD of triplicate samples from one experiment and are representative of four independent experiments. AU: arbitrary units. Concentrations of IFNβ and IL-8 in cell-culture supernatants were measured 24 h after stimulation. shMDA-5 and shIPS-1 THP-1 cells produced significantly less IFNβ and IP-10 mRNA and protein than control cells as measured 24 h post-infection (A and B) (*p*<0.05).

### Crosstalk between TLR2-MyD88 and the NALP3 inflammasome for IL-1β expression and processing

IL-1β is a key cytokine of antimicrobial host defenses, whose expression is regulated at a transcriptional and post-transcriptional level [36]. IL-1β is likely to play an important role during poxvirus infection, as suggested by the fact that poxviruses encode for IL-1β decoy receptor and disrupt intracellular IL-1 receptor signalling [37],[38]. We therefore examined whether activation of the TLR2-MyD88 pathway was implicated in the activation of the *IL1b* gene. As shown in Figure 8A, up-regulation of IL-1β mRNA was markedly impaired in TLR2^−/−^ and MyD88^−/−^ BMDMs infected with MVA, indicating that activation of the TLR2-MyD88 signalling pathway is critical for transcription of the *IL1b* gene during MVA infection. Secretion of mature IL-1β p17 in response to endogenous and exogenous danger signals requires the cleavage of the inactive pro-IL-1β precursor by the cysteine protease caspase-1. Conversion of pro-caspase-1 into caspase-1 is tightly regulated by the NALP3 inflammasome composed of NALP3, ASC and pro-caspase-1 [22]. To examine the contribution of the NALP3 inflammasome in the production of IL-1β triggered by MVA, we analyzed the expression of pro-IL-1β and IL-1β p17 in THP-1 cells deficient in NALP3, ASC or caspase-1 [39]. Knocking down of either one of the three components of the NALP3 inflammasome (i.e. NALP3, ASC or caspase-1) was associated with a massive reduction of mature and secreted IL-1β (Figure 8B and C). Similar results were obtained in THP-1 cells infected with NYVAC (Figure S1) and in NALP3^−/−^ BMDMs infected with MVA (Figure 8D and E). Of note, in THP-1 cells and in BMDMs the expression of pro-IL-1β was unaffected by the absence of either NALP3, ASC or caspase-1 clearly indicating that NALP3 inflammasome does not itself regulate the transcriptional and translation control of the IL-1β precursor. The NALP3 inflammasome was also dispensable for activation of the IRF3 transcription factor and IFNβ secretion (Figure S6). Altogether, these data demonstrate that IL-1β production after MVA infection requires a crosstalk between TLR2-MyD88 (initiation of the transcription and translational of IL-1β) and the NALP3 inflammasome (processing of pro-IL-1β into mature IL-1β).

**Figure 8:** Crosstalk between TLR2-MyD88 and the NALP3 inflammasome for IL-1β expression and processing. (A) Wild-type, TLR2^−/−^ and MyD88^−/−^ BMDMs were primed overnight with ultra-pure LPS (100 ng/ml) and infected with MVA (MOI 5). IL-1β mRNA expression was quantified by RT-PCR (*p*<0.05 for TLR2^−/−^ or MyD88^−/−^ *vs.* wild-type BMDMs). THP-1 cells stably transduced with control, NALP3, ASC and caspase 1 (casp1) shRNAs were infected with MVA (MOI 5 unless specified otherwise) for the indicated time (B–C). (B) Western blots of intracellular pro-IL-1β and secreted IL-1β p17. (C) IL-1β concentrations measured by ELISA in cell-culture supernatants collected 24 h after infection (*p*<0.05 for cells transduced with NALP3, ASC and casp1 shRNAs *vs.* control shRNA). LPS-primed wild-type and NALP3^−/−^ BMDMs were infected with MVA (MOI 5 in D) for 6 h (D–E). (D) Western blots of intracellular pro-IL-1β and secreted IL-1β p17. (E) IL-1β concentrations measured by ELISA in cell-culture supernatants collected 24 h after infection. Results are expressed as the ratio of IL-1β mRNA levels to that of HPRT. Data are means±SD of triplicate samples from one experiment and are representative of two independent experiments (*p*<0.05 for NALP3^−/−^ *vs.* wild-type BMDMs).

### MVA activates the NF-κB, ERK1/2, JNK, IRF3, IRF7 and STAT-1 signalling pathways

Poxviruses have been reported to activate the NF-κB, ERK1/2 and JNK pathways in epithelial and fibroblastic cell lines [40]–[43] and IRF3 and IRF7 in dendritic cells [24],[25]. Having identified the pathogen recognition receptors implicated in macrophage response to MVA (TLR2-TLR6, MDA-5 and NALP3), we next examined which downstream signalling pathways are activated for the expression of cytokines, chemokines and type I IFNs. Kinetics studies of NF-κB, ERK1/2 and JNK MAP kinases and IRFs activation were performed in THP-1 cells (Figure 9A). Electrophoretic mobility shift assay revealed that NF-κB nuclear content peaked 3 h after MVA infection. Phosphorylation of the ERK1/2 and JNK MAP kinases was between 1 and 6 h after infection. IRF3, which is essential for transcription of the *IFNB* gene, was detected 3 h after infection, peaked at 6 h and rapidly decreased thereafter. IRF7 was detected 3 h after infection and levels remained unchanged for 24 h. Phosphorylation of signal transducer and activator of transcription 1 (STAT-1), a critical target of IFNβ signalling required for the transcriptional activation of IFNβ-dependent genes, was first detected 3 h post-infection and gradually increased until 24 h (Figure 9A). The functional significance of the increased binding activity of NF-κB and phosphorylation of the IRF3 was confirmed by showing that MVA increased the transcriptional activities of multimeric-κB and IRF3-dependent-IFNβ promoter luciferase reporter vectors in transiently transfected THP-1 cells (Figure 9B and C). Confirming the importance of NF-κB and ERK1/2 in mediating innate immune response to MVA infection, pre-incubation of THP-1 cells with drugs (i.e. NEMO and U0126, see *Materials and Methods*) selectively inhibiting the NF-κB and ERK-1/2 signalling pathways impaired, albeit to a different extent, IL-1β (70% and 65% inhibition), IL-8 (75% and 72% inhibition) and IFNβ (28% and 42% inhibition) mRNA expression (*p*<0.05 for all conditions). Therefore, consistent with the fact that several pattern recognition receptors are engaged in the sensing of MVA by the innate immune system, multiple intracellular signalling pathways, including NF-κB, MAP kinases and IRFs were found to be activated upon infection of THP-1 macrophages with MVA. Of note, NYVAC induced very weak induction of intracellular signalling (i.e. NF-κB, ERK-1/2, IRF3 and STAT-1) and low levels of cytokines and IFNβ when compared with MVA (Figure S1) which is likely due to the expression of different patterns of immunomodulatory genes by these two poxviruses [24],[25].

**Figure 9:** MVA activates the NF-κB, ERK1/2, JNK, IRF3, IRF7 and STAT-1 signalling pathways. Electrophoretic mobility shift assay of NF-κB DNA binding activity and Western blots of phosphorylated ERK1/2 (P-ERK1/2), JNK (P-JNK), IRF3 (P-IRF3) and STAT-1 (P-STAT-1) and total ERK1/2, JNK and IRF7 (A). Nuclear (NF-κB) and cytosolic (ERK1/2, JNK, IRF3, IRF7, STAT-1 and tubulin) extracts were prepared from THP-1 cells infected with MVA (MOI 5) for the indicated time. Results are representative of three independent experiments. The retarded complex detected by EMSA was dose-dependently inhibited by cold wild-type but not mutant NF-κB oligonucleotide, and supershifted using anti-p65 antibody (data not shown). NF-κB- (B) and IRF3- (C) mediated transcriptional activities measured in THP-1 cells transiently transfected with trimeric κB sites or IRF3-dependent IFNβ promoter luciferase reporter vectors and infected with MVA (MOI 5 and 20) for 18 h. Results are expressed as the ratio of luciferase activity to *Renilla* luciferase activity. Data are means±SD of triplicate samples from one experiment and are representative of four independent experiments. *p* = 0.05, 0.02, 0.04 and 0.02 for MVA-infected (MOI 5 and 20) *vs.* control cells.

## Discussion

Analyses of pattern recognition receptors engagement by poxviruses are essential for improving our understanding of the pathogenesis of this important class of DNA viruses and for designing new viral vaccine vectors with improved immunogenicity. Dissection of the molecular bases of innate immune responses elicited by the attenuated poxvirus MVA strain in human macrophages revealed a critical role for TLR2-TLR6-MyD88, MDA-5-IPS-1 and NALP3 inflammasome pathways in the production of chemokines, IFNβ and IL-1β. These observations provide novel information on MVA recognition by sentinel innate immune cells and highlight the existence of potential differences between attenuated and non-attenuated poxviruses in the engagement of or recognition by innate sensors.

Up to now the retinoic acid-inducible gene-I-like receptors (RLR) RIG-I and MDA-5 had been viewed as master cytosolic sensors of RNA viruses [29]. However, recent observations suggested a role for the RLR pathway in the recognition of DNA viruses. Mouse embryo fibroblasts deficient in IPS-1 displayed reduced induction of IFNβ in response to MVA lacking the E3 protein [44]. Adenovirus and HSV1 have also been shown to replicate at much higher titers in RIG-I mutant than in RIG-I wild-type human hepatoma cell lines [45]. Moreover, microarray analyses revealed that RIG-I and MDA-5 expression was upregulated in human monocyte-derived dendritic cells infected with MVA [24]. Here we also showed that MVA caused a strong up-regulation of RIG-I, MDA-5 and IPS-1, yet only MDA-5 and IPS-1 were found to mediate MVA-induced IFNβ and IFNβ-dependent chemokine production by macrophages (Figure 10). As anticipated, transcriptional activation of *IFNb* and *IFNb-dependent* chemokine genes was associated with the activation of IRF3 and IRF7 and STAT-1. To the best of our knowledge this is the first demonstration of a direct role for MDA-5 in innate sensing of a DNA virus. Moreover, the MDA-5/IPS-1 pathway was also implicated in the production of IFNβ by macrophages infected with the NYVAC and the Western Reserve strains of vaccinia virus (Figure S1 and S2).

**Figure 10:** Pathways activated by MVA in the macrophage. Infection of macrophages with MVA stimulates the TLR2-TLR6-MyD88, MDA-5/IPS-1 and NALP3 inflammasome pathways leading to the activation of NF-κB, ERK-1/2, JNK, IRF3, IRF7 and STAT-1 that are involved in the transcriptional activation of genes encoding for cytokines, chemokines and type I IFN. At the cell surface, MVA is sensed by the TLR2-TLR6 heterodimer that induces the production of IFNβ-independent chemokines (IL-8, MIP-1 and MIP-2) (1) and pro-IL-1β (2). Upon virus entry into the cell, cytosolic MVA or MVA-derived viral components (possibly envelope or core proteins, early mRNA or DNA) activate the MDA-5-IPS-1 pathway to release IFNβ (3) and subsequent induction of IFNβ-dependent chemokines (such as RANTES, IP-10) following activation of the type I IFN receptor (4). Finally, MVA infection leads to the activation of the NALP3 inflammasome (composed of NALP3, ASC and pro-caspase 1) enabling caspase-1 processing, pro-IL-1β maturation and IL-1β secretion (5). For simplicity, the same diagram for MVA is shown outside and inside the cell.

RIG-I has been shown to be involved in the induction of TNF and type I IFN by myxoma poxvirus in human macrophages [46]. Yet, silencing of MDA-5 was associated with a small (about 25%) but clear reduction of macrophages response to myxoma virus suggesting that both RIG-I and MDA-5 were implicated, albeit to various degree, in innate immune response to myxoma virus. The nature of the component(s) of DNA viruses activating the RLR pathway remains to be identified. Obvious candidate molecules include, envelope or core proteins, early mRNA and DNA itself. Unless RLR engagement is used primarily to the virus own benefit, it is likely that poxviruses have developed antiviral escape strategies interfering with the host RLR antiviral defense pathway. In line with this assumption, the dsRNA binding protein E3 of vaccinia virus has been reported to inhibit IPS-1 signaling, IRF3 phosphorylation, cytokine and IFNβ production [47]–[49]. Should inhibitors of the RLR pathway be identified in the MVA genome, gene deletion might provide an opportunity to generate new MVA vaccine vectors with increased immunogenicity.

In addition to RLR, profiling of the cytokine response induced by MVA in the macrophage revealed a key role for the heterodimeric TLR2-TLR6 complex and the adapter protein MyD88 in the production of IFNβ-independent chemokines (such as IL-8, MIP-1α, MIP-1β and MIP-2) (Figure 10). Innate immune recognition of the vaccinia virus has also been shown to depend on TLR2 and MyD88 [32]. The present observation is one of the few examples of viral recognition mediated by TLR2 heterodimers. Recognition of human cytomegalovirus has been shown to be mediated by a TLR2-TLR1 heterocomplex and that of hepatitis C virus by either TLR2-TLR1 or TLR2-TLR6 [50],[51]. The facts that TLR2 is expressed at the cell surface and that the inhibition of endocytosis or UV-irradiation of MVA did not affect IL-8 production by macrophage suggest that a component of the MVA envelope or a core protein is responsible for the activation of the TLR2-TLR6-MyD88 pathway. However, the nature of the viral component likely to serve as ligands for these TLR2-TLR1/TLR6 heterodimers has so far remained elusive.

Other TLRs have also been implicated as innate sensors of poxviruses. Ectromelia virus, the causative agent of mousepox, was shown to be recognized by mouse dendritic cells in TLR9 dependent manner [33]. In contrast, responses of dendritic cells to MVA was both TLR9-dependent (up-regulation of CD40) and TLR9-independent (up-regulation of CD69 and production of IFNα and IL-6) [33],[52]. Although we did not perform experiments with TLR9-deficient macrophages in the present study, the data obtained with MyD88 deficient cells clearly rule out the implication of TLR9 in MVA-induced IFNβ and IFNβ-dependent chemokines. However, we cannot exclude the involvement of TLR9 in the production of IFNβ-independent chemokines. Finally, in a mouse model activation of TLR3 contributed to the pathogenesis of Western Reserve vaccinia virus [53]. In contrast, experiments conducted with TRIF-deficient macrophages clearly showed that the production of chemokines and IFNβ induced by MVA was TLR3-independent in the present study. Taken together these observations demonstrate that TLRs may exert a two-sided role in poxvirus infections acting on the one hand as key initiators of the host anti-poxvirus defense response and on the other hand as important mediators of viral pathogenicity and tissue damage.

The other important intracellular innate immune sensor of microbial products and endogenous molecules is the NALP3 inflammasome that controls the processing and maturation of the cytokines IL-1β and IL-18 [22]. Here we show that MVA is a potent activator of the NALP3 inflammasome and of IL-1β release by macrophages. IL-1β and IL-18 are key mediators of the host antimicrobial defense response and several lines of evidence suggest that these cytokines are likely to play an important role in host defenses against poxvirus infections. For example, the *B15R* gene of the vaccinia virus encodes an IL-1β decoy receptor blocking the activity of IL-1β and IL-18 and inactivation of *B15R* gene reduces the virulence of the vaccinia virus [38],[54]. Furthermore, poxviruses release IL-18 binding proteins inhibiting IL-18 activity and vaccinia viruses *A46R*, *A52R*, *N1L* and, *K1L* gene products have been shown to disrupt the IL-1 receptor intracellular signaling pathway at multiple levels [37],[55]. Interestingly, we observed that MVA stimulated the release of large amounts of the IL-1 receptor antagonist by macrophages (Figure 3C) adding further support to the view that IL-1 is an important target of the poxvirus antiviral escape strategy. Finally, consistent with the notion that the NALP3 inflammasome plays an important role in host defenses against poxviruses, several inhibitors of caspase-1 and ASC, like CrmA (cowpox virus), M13L-PYD (myxoma virus) and PYD-only (shope fibroma-virus) have been identified in the genomes of several poxviruses [56]–[58].

Crosstalks between TLRs and NLRs have been demonstrated to occur in the course of bacterial infections, such as between TLR5 and the IPAF inflammasome after exposure to flagellated bacteria or the flagellin protein itself [59]–[61]. To the best of our knowledge, however, the present data provide the first demonstration of a crosstalk between the TLR and NLR pathways in the context of a viral infection (Figure 10). While TLR2 and MyD88 were necessary to induce IL-1β mRNA expression (Figure 8A), the NALP3 inflammasome was absolutely required for the processing of pro-IL-1β and IL-1β secretion (Figure 8B and C). Dual activation pathways coupling MVA recognition to IL-1β may provide the host with an increased capacity of fine tuning of its cytokine response.

In summary, the present data show that the TLR2-TLR6-MyD88, MDA-5-IPS-1 and NALP3 inflammasome pathways exert both specific and coordinated functions in the sensing of MVA infection and in the regulation of cytokine, chemokine and IFNβ responses (Figure 10). After the unfortunate failure of the adenovirus type 5 HIV vaccine STEP trial due to issues related to natural immunity against this virus, the attenuated MVA and NYVAC strains of poxvirus have become attractive vaccine vectors against HIV/AIDS. Arguments supporting the use of MVA and NYVAC as vaccine vectors include excellent immunogenicity and safety profiles and limited pre-existing immunity to poxvirus in the population at risk of HIV infection due to the abandon of vaccine campaigns after the eradication of smallpox in the 1970s. The present findings are therefore likely to provide important information relevant to the study of the pathogenesis of poxvirus infections, the understanding of antiviral escape mechanisms of poxvirus and may help to design new vaccine vectors with increased immunogenicity.

## Materials and Methods

### Ethics statement

All animal procedures were approved by the Office Vétérinaire du Canton de Vaud (authorizations n° 876.5, 876.6, 877.5 and 877.6) and performed according to our institution guidelines for animal experiments.

### Mice

Eight to ten-week-old female BALB/c and C57BL/6 mice were purchased from Charles River Laboratories (L'Arbresle, France) and were acclimatized for at least one week before experimentation. MyD88^−/−^, TRIF^−/−^, TLR1^−/−^, TLR2^−/−^, TLR4^−/−^, TLR6^−/−^ and NALP3^−/−^ C57BL/6 mice have been described previously [62]–[68]. Mice were bred and housed in specific pathogen free conditions.

### Cells and reagents

The human monocytic THP-1 cell line (American Type Culture Collection, Manassas, VA) was cultured in RPMI 1640 medium containing 2 mM L-glutamine, 50 µM 2-mercaptoethanol, 100 IU/ml of penicillin, 100 µg/ml of streptomycin (all from Invitrogen, San Diego, CA) and 10% heat-inactivated FCS (Sigma-Aldrich, St. Louis, MO). THP-1 cells differentiated into macrophages by treatment with 0.5 mM phorbol 12-myristate 13-acetate (PMA, Sigma-Aldrich) for 24 h were used in all experiments except those for reporter gene analyses. THP-1 cells stably expressing control, NALP3, caspase-1 and ASC shRNA have been described previously [69],[70]. THP-1 cells expressing TLR2, IPS-1, MDA-5 and RIG-I shRNA were generated using lentiviruses expressing hairpins directed against TLR2, IPS-1 and MDA-5 (5 for TLR2, 5 for IPS-1, 2 for MDA-5 and 5 for RIG-I) produced with the second-generation pMD2-VSVG and pCMV-R8.91 packaging plasmids as described previously and cultured in the presence of 5 µg/ml puromycin [71]. The sequence of the hairpins selected that gave the best targeting of TLR2, IPS-1, MDA-5 and RIG-I were AAACCCAGGGCTGCCTTGGAAAAG, CAAGTTGCCAACTAGCTCAAA, CCAACAAAGAAGCAGTGTATA and AAACCCAGGGCTGCCTTGGAAAAG, respectively. Levels of expression of targeted genes were analyzed by real-time PCR using specific oligonucleotides (Table S1) and the most efficiently silenced THP-1 subsets were selected for further studies (*i.e.* cell lines #1 in Figure S2).

Peripheral blood mononuclear cells from healthy donors (recruited by the Blood Center, Lausanne, Switzerland) were purified by Ficoll-Hypaque density gradient (GE Healthcare, Uppsala, Sweden). Macrophages were obtained by culturing adherent PBMCs cells for 6 days in RPMI 1640 with Glutamax. Bone marrow-derived macrophages (BMDMs) isolated from wild-type, TLR1^−/−^, TLR2^−/−^, TLR4^−/−^, TLR6^−/−^, MyD88^−/−^ and TRIF^−/−^ mice were cultured for 7 days in IMDM (Invitrogen) containing 50 µM 2-mercaptoethanol and monocyte-colony stimulating factor to obtain BMDMs. All media were supplemented with 10% FCS, 100 IU/ml of penicillin and 100 µg/ml of streptomycin. In selected experiments, cells were stimulated with 100 ng/ml *Salmonella minnesota* ultra pure LPS (List Biologicals Laboratories, Campbell, CA), 10 µg/ml polyinosine-polycytidylic acid (poly(I∶C), Invivogen, San Diego, CA), 1–10 µg/ml S-[2,3-bis(palmitoyloxy)-(2RS)-propyl]-[R]-cysteinyl-[S]-seryl-[S]-lysyl-[S]-lysyl-[S]-lysyl-[S]-lysine×3 CF3COOH (Pam_2_CSK_4_) or N-Palmitoyl-S-[2,3-bis(palmitoyloxy)-(2RS)-propyl]-[R]-cysteinyl-[S]-seryl-[S]-lysyl-[S]-lysyl-[S]-lysyl-[S]-lysine×3 HCl (Pam_3_CSK_4_) lipopeptides (EMC microcollections, Tuebingen, Germany), or treated with 50 µg/ml of anti-IFNβ antibodies (BioLegend, San Diego, CA), 2 µM cytochalasine D, 100 µM chloroquine (Sigma-Aldrich), 10 µM SB203580 (p38 inhibitor), 10 µM U0126 (MEK1/2 inhibitor) or 50 µg/ml NEMO-binding domain binding peptide (IkB kinase inhibitor) (Calbiochem-Novabiochem, Nottingham, UK).

### MVA, NYVAC and WR production, *in vitro* and *in vivo* models of infection

MVA and NYVAC were cultured in chicken embryo fibroblasts and WR in HeLa cells. Viruses were purified by two sucrose cushions and titrated on BHK-21 and BSC-40 cells as previously described [24],[72]. Cells were infected with MVA, NYVAC or WR at various multiplicities of infection (MOI 1, 5 or 20 pfu/cell). After 1 h of contact with cells, the virus inoculum was removed and fresh medium added to the cultures. Cell-culture supernatants and cells were collected at different time points after infection and processed for flow cytometry, Luminex technology, ELISA, RNA extraction, and Western blot analyses. In selected experiments, MVA suspension (0.2 ml in 24-well plates laid on ice) was irradiated by a 15-min exposure to a 365-nm UV bulb at a distance of 4 cm. UV-irradiation caused a 90% inhibition of the expression of C6L early gene as determined by RT-PCR using oligonucleotides (5′-3′ sense and antisense at position −19541/−19503 and −19071/−19090 in MVA019L) AACTGCAGAAATGAATGCGTATAATAAAGCCGATTCGTTTTCTTTAGAG and CGGGATCCTTACTTGTCATCGTCGTCGTTCTTGTAGTCCSTGTTTAGGAAAAAAfAAATATC. MVA did not propagate in THP-1 cells as demonstrated by the absence of infective viral particles in cell-culture supernatants collected 24 h after infection (data not shown).

For whole blood assay, 100 µl of heparinized whole blood collected from 3 healthy volunteers were diluted 5-fold in RPMI 1640 medium containing MVA (MOI 1) and incubated for 24 h at 37°C in the presence of 5% CO_2_. Samples were centrifuged, and cell-free supernatants were stored at −80°C until cytokine measurement. For *in vivo* studies, 2×10^7^ PFU of MVA in 1 ml phosphate-buffered saline (PBS) were injected intraperitoneally into BALB/c mice. After 12 h, a peritoneal lavage was performed. The supernatant obtained after centrifugation of the lavage fluid was collected for cytokine measurement by ELISA whereas the cell pellet was processed for gene expression analysis by RT-PCR. Spleens were collected from the same animals to quantify cytokine protein and mRNA expression levels.

### Flow cytometry

To follow cell infection, THP-1 cells were infected (MOI 5) with a GFP-expressing mutant MVA, whereas all other experiments used wild-type MVA. The percentage of GFP-positive THP-1 cells was measured 0, 2, 4, 6, 12 and 24 h after infection. MVA-induced cell apoptosis was determined 6 h and 24 h post-infection using the Annexin-V FITC apoptosis detection kit according to manufacturer's recommendations (BD Biosciences, Erembodegem, Belgium). Acquisition and analysis were performed using a FACS Calibur (BD Biosciences) and FlowJo 8.5.3 software (FlowJow, Ashland, OR).

### Measurement of cytokine production

A screening of mediators produced by MVA-infected THP-1 cells was performed with the human cytokine Bioplex assay (Bio-Rad, Hercules, CA) using the Luminex technology (Luminex Corporation, Austin, TX) available at the Cardiomet Mouse Metabolic Evaluation Facility, Center for Integrative Genomics, University of Lausanne, Lausanne, Switzerland. Thirty mediators were tested: TNFα, IL-1α, IL-1ra, IL-1β, IL-2, IL-4, IL-5, IL-6, IL-7, IL-8, IL-10, IL-12p40, IL-12p70, IL-13, IL-15, IL-17, IFNγ, RANTES, IP-10, MIP-1α, MIP-1β, MCP-1, eotaxin, fractalkine, TGFα, EGF, VEGF, GM-CSF, G-CSF and sCD40L. The concentrations of human IL-1β (Bender MedSystems, Vienna, Austria), IL-8, (BD Biosciences), IP-10, MIP-1α (R&D) and IFNβ (PBL Biomedical Laboratories, Picataway, NJ) in whole blood assay and cell-culture supernatants were measured by ELISA. TNF and IL-6 concentrations were measured by bioassay as described elsewhere [73]. Mouse IL-1β, MIP-2 (R&D) and IFNβ were quantified by ELISA (Biomedical Laboratories, Picataway, NJ).

### RNA analysis by quantitative real-time polymerase chain reaction

Total RNA was isolated from THP-1 cell lines, human monocytes/macrophages, peritoneal cells and splenocytes using the RNeasy kit (Qiagen, Hombrechtikon, Switzerland). Reverse transcription of 1 µg of RNA was performed using the ImProm II RT System kit (Promega, Dübendorf, Switzerland). Quantitative PCR was performed with a 7500 Fast Real-Time PCR System (Applied Biosystems, Rotkreuz, Switzerland) using the Power SYBR Green PCR Master Mix (Applied Biosystems) and primer pairs listed in Table S1. All samples were tested in triplicates. Amplifications consisted of a denaturation step at 95°C for 15 sec and an annealing/extension step at 60°C for 60 sec, with the 9600 Emulation mode. For each measurement, a standard made of successive dilutions of a reference cDNA was processed in parallel. Gene specific expression was expressed relative to the expression of *HPRT* in arbitrary units (A.U.). Gene specific over *HPRT* ratios were validated using the house-keeping gene *ACTB* (human studies) or *Gapdh* and *Actg1* (mouse studies).

### Transfection and reporter assay

THP-1 cells were seeded at 5×10^4^ cells per well in 24-well plates. The following day, cells were transiently transfected with 700 ng of multimeric κB site [73] and IFNβ promoter [74] luciferase reporter vectors together with 70 ng of a *Renilla* luciferase control vector (Promega) using jetPEI™ transfection reagent (Polyplus-transfection SA, Illkirch, France). Twenty-four h after transfection, cells were infected with MVA. Luciferase and *Renilla* luciferase activities were measured 24 h latter using the Dual-LuciferaseTM Reporter Assay System (Promega). Results were expressed as relative luciferase activity (the ratio of luciferase to *Renilla* luciferase activity).

### Western blot analysis

THP-1 cells were washed with ice cold PBS and lysed for 5 min at 4°C with the M-PER Mammalian Protein Extraction Reagent (Pierce Biotechnology Inc, Rockford, IL). Reaction mixtures were centrifuged 5 min at 14'000 rpm. Protein concentration of supernatants was determined using the bicinchoninic acid protein assay (Pierce Biotechnology). Cell-lysates were electrophoresed through 12% (w/v) polyacrylamide gels and transferred onto nitrocellulose membranes (Schleicher & Schuell, Keene, NH). Membranes were incubated with antibodies directed against RIG-1, MDA-5, IPS-1 (Apotech Corporation, Epalinges, Switzerland), cleaved IL-1β, total- and phospho-p44/42 (ERK1/2), and -JNK MAP Kinases, phospho-IRF3 (Cell Signalling Technology, Danvers, TX), caspase 1 (Santa Cruz, Santa Cruz, CA), phospho-STAT-1 (BD Biosciences), IRF7 (Zymed, San Franciso, CA) and tubulin (Sigma). After washing, membranes were incubated with horse radish peroxidase (HRP)-conjugated secondary antibody (Pierce). Signals were revealed using the ECL Western blotting Analysis System (GE Healthcare).

### Electrophoretic mobility shift assay (EMSA)

Nuclear extracts were prepared and analyzed by EMSA [73]. Briefly, protein concentration of cell extracts was measured using the Bradford-dye assay (Bio-Rad). Two µg of nuclear extracts were incubated for 15 min at room temperature with a radio-labeled consensus NF-κB probe (Santa Cruz). Reaction mixtures were electrophoresed through 6% non-denaturing polyacrylamide gels. Gels were dried and exposed to X-ray films. Supershift experiments using anti-p65 antibody (sc-109, Santa Cruz) were performed as previously described [75] (data not shown).

### Statistical analyses

Comparisons among treatment groups were performed by two-tailed paired Student's *t*-test. *p* values less than 0.05 were considered to indicate statistical significance.

## Supporting Information

Figure S1 Comparison of macrophage responses to MVA and NYVAC. THP-1 cells (A, B, D, F) and THP-1 cells stably expressing control, TLR2, MDA-5, RIG-I, IPS-1, NALP3 and caspase-1 shRNAs (C, E) were infected with MVA and NYVAC (MOI 5). Cytokines, chemokines and IFNβ production were assessed by ELISA (A, E). IL-8, IFNβ, IP-10, MIP-1α and RANTES mRNA levels were analyzed by RT-PCR and expressed as reported in Figure 1 (B, C). Electrophoretic mobility shift assay of NF-κB DNA binding activity and Western blot analyses of RIG-I, MDA-5, IPS-1, phosphorylated ERK1/2 (P-ERK1/2), IRF3 (P-IRF3) and STAT-1 (P-STAT-1) and tubulin (D, F). Data are means±SD of triplicate (A, B, C, E) samples from one experiment and are representative of two to three independent experiments. ND: not detected (A).
(0.12 MB PDF)

Figure S2 TLR2 and MDA-5 contribute to the production of IL-8 and IFNβ by human macrophages infected with the Western Reserve strain of vaccinia (WR). THP-1 cells (A–B) and THP-1 cells stably expressing control, TLR2, MDA-5, RIG-I and IPS-1 shRNAs (C) were infected with WR (MOI 5). IL-8 and IFNβ mRNA levels were analyzed by RT-PCR and expressed as reported in Figure 1 (A and C). IL-8 and IFNβ production by THP-1 cells stimulated for 24 h with WR were assessed by ELISA (B). Data are means±SD of triplicate samples from one experiment and are representative of two independent experiments. shTLR2 THP-1 cells produced significantly less IL-8, whereas shMDA-5 and shIPS-1 THP-1 cells produced significantly less IFNβ than control cells (C) (*p*<0.05).
(0.02 MB PDF)

Figure S3 TLR2 contributes to the production of IFNβ-independent chemokines by THP-1 macrophages infected with MVA. THP-1 cells stably expressing control and candidate shRNA (#1 and #2) directed against TLR2 were obtained as described in *Materials and Methods*. (A) TLR2 mRNA content was analyzed by RT-PCR. Results are expressed as the ratio of TLR2 mRNA levels to that of HPRT. (B) shControl and shTLR2 THP-1 cells were infected with MVA (MOI 5 unless specified) or stimulated with Pam_3_CSK_4_ (1 µg/ml) for 24 h unless otherwise specified. IL-8, MIP-1α, IFNβ and IP-10 mRNA contents were analyzed by RT-PCR. Results are expressed as the ratio of IL-8, MIP-1α, IFNβ and IP-10 mRNA levels to that of HPRT. (C) IL-8 concentrations were measured by ELISA. Data are means±SD of triplicate samples from one experiment and are representative of three (A, B) or two (C) independent experiments. AU: arbitrary units. shTLR2 THP-1 cells produced significantly less IL-8 and MIP-1α mRNA (B) and IL-8 protein than control cells (C) (*p*<0.05).
(0.02 MB PDF)

Figure S4 MVA infection increases RIG-I and MDA-5 mRNA expression *in vivo*. BALB/c mice were injected i.p. with MVA (10^7^ PFU). Peritoneal cells (A) and splenocytes (B ) were isolated 12 h after infection as described in *Materials and Methods*. RIG-I and MDA-5 mRNA contents were analyzed by RT-PCR. Results are expressed as the ratio of RIG-I and MDA-5 mRNA levels to that of HPRT. AU: arbitrary units. Data are means±SD of triplicate samples from one experiment comprising three mice per experimental condition and are representative of two independent experiments (*p*<0.05 for all conditions).
(0.01 MB PDF)

Figure S5 Generation of THP-1 cells expressing reduced levels of RIG-I, MDA-5 and IPS-1. THP-1 cells stably expressing control and candidate shRNA (#1 and #2) directed against RIG-I, MDA-5 and IPS-1 were obtained as described in *Materials and Methods*. RIGI, MDA-5 and IPS-1 mRNA contents were analyzed by RT-PCR and expressed as reported in Figure 1. Data are means±SD of triplicate samples from one experiment and are representative of two independent experiments.
(0.01 MB PDF)

Figure S6 The NALP3 inflammasome is dispensable for activation of the IRF3 transcription factor and IFNβ secretion. THP-1 cells stably expressing control, NALP3, ASC and caspase 1 (casp1) shRNAs were infected with MVA (MOI 5 unless specified otherwise) (A, B) or cultured with (+) or without (−) monosodium urate monohydrate (MSU) cristals crystals for the indicated time (A) or 6 h (B, C). Western blots of intracellular phosphorylated IRF3 and tubulin (A) and IFNβ (B) and IL-1β (C) concentrations measured by ELISA in cell-culture supernatants. Data are means±SD of triplicate samples from one experiment and are representative of two independent experiments. *p*<0.05 for cells transduced with NALP3, ASC and casp1 shRNAs *vs.* control shRNA (C).
(0.12 MB PDF)

Table S1 Oligonucleotides used in RT-PCR analyses.
(0.02 MB PDF)
